# A Complex Case of Dysmenorrhea and Concurrent Acute Appendicitis

This article has been retracted.

**DOI:** 10.7759/cureus.8734

**Published:** 2020-06-21

**Authors:** Ahmed Elkhouly, Mohab Hassib, Talha Awwal, Anand Kaji

**Affiliations:** 1 Internal Medicine, St. Francis Medical Center, Trenton, USA

**Keywords:** dysmenorrhea, appendicitis, cyclic vomiting

## Abstract

Dysmenorrhea is a common problem experienced by many women on a regular basis. It is characterized by recurrent bouts of crampy abdominal pain that is associated with the menstrual cycle. These episodes can vary in severity and frequency and may require treatment. The objective of this study is to shed light on a case of severe dysmenorrhea that occurred simultaneously with acute appendicitis. The patient underwent appendectomy, but despite this continued to have abdominal pain in the postoperative period. This led to many investigations for possible post-surgical complications that had no yield. The diagnosis of dysmenorrhea was made with help from family members who disclosed that the patient had heavy bleeding and severe crampy menstrual pain associated with nausea and vomiting. This information was unknown to the medical team as this patient did not disclose this information. The coincidence of dysmenorrhea and concurrent acute appendicitis led to difficulty in diagnosing the etiology of the lingering postoperative abdominal pain.

## Introduction

Dysmenorrhea is the most common gynecological problem in menstruating females [1]. It is a significant medical issue that commonly results in absence from work or school. The annual monetary loss due to absences is estimated in the billions of US dollars [1]. Dysmenorrhea presents with variable severity and occurs before and/or during their menstrual period. Although pain can be a subjective experience, surveys of women have shown that more than 90% of women of reproductive age experience some form of dysmenorrhea [1]. Dysmenorrhea can be subdivided into primary and secondary dysmenorrhea. Primary dysmenorrhea is characterized as painful menstruation with no identifiable causes, whereas secondary dysmenorrhea is painful menstruation due to an established pelvic pathology.

Primary dysmenorrhea is described as premenstrual and peri-menstrual pain in the absence of other precipitating factors. The onset of primary dysmenorrhea is usually within the first three years of menarche but typically not within the first six months [2]. Women with primary dysmenorrhea often have increased endometrial prostaglandin production that leads to increased uterine tone and stronger uterine contractions which manifests as pain [1,3]. Females with more painful menstrual cycles are found to have higher levels of PGF2a in their menstrual fluid [1]. Nonsteroidal anti-inflammatory medications and oral contraceptive pills (OCPs) are the treatments of choice, although 10% of affected females find no relief with these treatments [1]. For patients who are resistant to these medications, further investigations should be carried out to rule out causes of secondary dysmenorrhea.

Secondary dysmenorrhea has comparable symptoms to the primary form of the disease; however, it is preceded by a pelvic pathology. The most common etiologies are endometriosis, fibroids, adenomyosis, and pelvic inflammatory disease. Some key differentiating characteristics of secondary dysmenorrhea are dyspareunia and resistance to treatment [1]. Secondary dysmenorrhea also displays a different temporality when contrasted with primary dysmenorrhea. In secondary dysmenorrhea, menstrual pain may begin in the first cycle following menarche or may occur later in life, around age 25, without any previous history of painful periods [1].

## Case presentation

A 20-year-old female patient with no past medical history presented to the emergency department with a one-day history of intractable bilious vomiting and diffuse abdominal pain. She describes the pain as sharp, diffuse, non-radiating, and severe to the extent that she had difficulty speaking and refused examination. She denied any sick contacts, recent travel, or ingestion of fast food prior to the vomiting commencing. A CT scan on admission showed bowel wall thickening and a dilated appendix with mild inflammation in the periappendiceal fat (Figure 1)*​​​​​​*. Her relevant laboratory findings were: a white blood cell count of 14.4 x 10^3^/uL with a neutrophilia of 81.8%, a lipase of 5 U/L, a lactate of 2.1 mmol/L, and a hemoglobin of 11.3 g/dL. Furthermore, her vital signs were within normal limits, her chest X-ray was normal, initial blood cultures showed no bacterial growth, and pregnancy test was negative.

**Figure 1:** CT scan of the abdomen showing acute appendicitis.

At that point, a surgical opinion was sought. The likely differentials were acute appendicitis and colitis. The patient was taken to the operating room on the same day for an appendectomy and exploratory laparoscopy, during which a dilated non-perforated long inflamed appendix was excised without complications. Day 1 post-operatively, the patient continued to have abdominal pain and intractable bilious vomiting. She coincidentally also started to have menstrual bleeding on this day and received multiple doses of Toradol to relieve the ongoing abdominal pain. A repeat CT scan showed suspected post-operative changes (Figure 2).

**Figure 2:** CT scan of the abdomen showing post appendectomy changes.

A gastroenterology opinion was sought as the bilious vomiting persisted for three days post-operatively. She was not able to advance her diet for several days due to ongoing nausea and vomiting. The patient had an endoscopic evaluation, which showed mild acute esophagitis and non-erosive gastritis in the body and fundus (Figure 3).

**Figure 3:** Upper endoscopy showing non-erosive gastritis and oesophagitis.

The patient spontaneously improved over the next two days. Her nausea and vomiting subsided gradually, she was able to advance her diet, and was discharged from the hospital.

## Discussion

The simultaneous occurrence of acute appendicitis and dysmenorrhea perplexed the diagnosis and led us to believe that the patient was having postoperative complications. At the time of presentation, this patient had classical signs and symptoms of acute appendicitis. The imaging increased the likelihood of acute appendicitis, displaying periappendiceal inflammation. Following laparoscopic appendicectomy, her bilious vomiting persisted, and we were unable to advance her diet for three days. At this stage a post-operative bowel perforation or iatrogenic uterine injury was suspected as the patient started to have vaginal bleeding that day. These differentials were ruled out by a repeat CT scan. Considering the continued bilious vomiting and a normal CT scan, the patient went for an endoscopy that only showed esophagitis and non-erosive gastritis which were likely secondary to repeated episodes of vomiting, and the etiology of her vomiting remained unclear.

Dysmenorrhea was suspected in a patient with vaginal bleeding and severe abdominal pain associated with bilious vomiting, where no other abnormalities were found. Another factor that complicated this case was the patient’s demeanor. She was unwilling to answer any questions and therefore very little medical history was obtained from the patient. The patient did not have any visitors or family present in the hospital, however, after one week, her mother came to visit her and we were able to ask her about the patient’s general health and habits, after obtaining the patient’s consent. Her mother revealed that the patient typically had nausea and intermittent vomiting for several days on a monthly basis that is usually related to her menstrual period. She also explained that the patient was given Ibuprofen and a trial of OCPs that improved her symptoms. With this new information, as well as a normal endoscopy and imagine studies, a diagnosis of dysmenorrhea was established.

The objective of treatment in dysmenorrhea is to improve symptoms by decreasing the number of circulating prostaglandins. Cyclooxygenase inhibitors, including nonsteroidal anti-inflammatory drugs (NSAIDs), lower the number of menstrual prostaglandins released which depresses uterine hypercontractility [4]. OCPs also decrease menstrual prostaglandins and inhibit endometrial development [4]; they can be used for those with dysmenorrhea requiring contraception. Although with OCPs, high doses are typically needed to control symptoms [5].

A novel therapy that is currently being explored is the use of Dienogest, a progesterone-only hormone therapy used in the treatment of endometriosis, for the treatment of primary dysmenorrhea. A randomized multi-center trial of Dienogest versus placebo showed superiority in pain control with the use of Dienogest [6]. Although this is a promising prospect, a study comparing the use of progesterone-only medication versus estrogen containing OCPs would be useful in establishing a recommendation for first-line therapy. Another therapy that can be beneficial and inexpensive, is the use of therapeutic exercise to better control symptoms of dysmenorrhea. A systematic review and meta-analysis showed that physical exercise resulted in an improvement in both intensity and duration of pain in those who suffer from dysmenorrhea. This study should be interpreted with care however, as the type of exercise that leads to these positive results is varied [7].

## Conclusions

This case of acute appendicitis was thought to be complicated by postoperative vaginal bleeding, abdominal pain, and bilious vomiting; however, the patient was experiencing symptoms of severe dysmenorrhea. This very common menstrual disease is characterized mainly by pain and varies widely in severity causing it to mimic other diseases and leads to expensive and unnecessary investigations. The diagnosis can be achieved by obtaining a thorough history, and symptoms are usually responsive to non-steroidal anti-inflammatory medications or OCPs which both lower prostaglandins, leading to decreased uterine contractility and improving menstrual pain.
